The article "Electroacupuncture Treats Myocardial Infarction by Influencing the Regulation of Substance P in the Neurovascular to Modulate PGI2/TXA2 Metabolic Homeostasis via PI3K/AKT Pathway: A Bioinformatics-Based Multiomics and Experimental Study" was retracted in 2023. Reasons: signs of a paper mill; compromised peer review; unreliable results or conclusions.

# Electroacupuncture Treats Myocardial Infarction by Influencing the Regulation of Substance P in the Neurovascular to Modulate PGI2/TXA2 Metabolic Homeostasis via PI3K/AKT Pathway: A Bioinformatics-Based Multiomics and Experimental Study

**DOI:** 10.1155/2022/5367753

**Published:** 2022-09-22

**Authors:** Ping Zhang, Yanyan Wang, Xiaomin Xing, Hu Li, Xiaojing Wang, Hanlin Zhang, Xin Wang, Xiubin Li, Yanju Li, Qian Wang

**Affiliations:** ^1^Department of Rehabilitation, The Second Affiliated Hospital of Shandong First Medical University, Taian, 271000, China; ^2^Taian Traffic Hospital, Taian, 271000, China; ^3^Department of Neurology, The Second Affiliated Hospital of Shandong First Medical University, Taian, 271000, China; ^4^Postdoctoral Workstation, Department of Central Laboratory, The Affiliated Taian City Central Hospital of Qingdao University, Taian 271000, China

## Abstract

Acute myocardial infarction (AMI) is the most severe form of coronary heart disease caused by ischemia and hypoxia. The study is aimed at investigating the role of neuropeptides and the mechanism of electroacupuncture (EA) in acute myocardial infarction (AMI) treatment. Compared with the normal population, a significant increase in substance P (SP) was observed in the serum of patients with AMI. PGI2 expression was increased in the SP-treated AMI mouse model, and TXA2 expression was decreased. And PI3K pathway-related genes, including *Pik3ca*, *Akt*, and *Mtor*, were upregulated in myocardial tissue of SP-treated AMI patients. Human cardiomyocyte cell lines (HCM) treated with SP increased mRNA and protein expression of PI3K pathway-related genes (*Pik3ca*, *Pik3cb*, *Akt*, and *Mtor*). Compared to MI control and EA-treated MI rat models, *Myd88*, *MTOR*, *Akt1*, *Sp*, and *Irak1* were differentially expressed, consistent with in vivo and in vitro studies. EA treatment significantly enriched PI3K/AKT signaling pathway genes within MI-associated differentially expressed genes (DEGs) according to Kyoto Encyclopedia of Genes and Genomes (KEGG). Furthermore, it was confirmed by molecular docking analysis that PIK3CA, AKT1, and mTOR form stable dockings with neuropeptide SP. PI3K/AKT pathway activity may be affected directly or indirectly by EA via SP, which corrects the PGI2/TXA2 metabolic imbalance in AMI. MI treatment is now better understood as a result of this finding.

## 1. Introduction

Acute myocardial infarction (AMI) is the most severe manifestation of coronary heart disease. More and more young people are suffering from AMI, one of China's most critical public health problems [1]. It is primarily caused by ruptured coronary atherosclerotic plaques, which activates the body's platelets and coagulation process, eventually leading to thrombosis and coronary artery blockage [2].

The article "Electroacupuncture Treats Myocardial Infarction by Influencing the Regulation of Substance P in the Neurovascular to Modulate PGI2/TXA2 Metabolic Homeostasis via PI3K/AKT Pathway: A Bioinformatics-Based Multiomics and Experimental Study" was retracted in 2023. Reasons: signs of a paper mill; compromised peer review; unreliable results or conclusions.

AMI causes ischemia and hypoxia in the myocardium, which can cause pain, anxiety, and changes in cardiac function and promote sympathetic nerve activity. Neuropeptides are important prognostic markers of AMI [3–6]. The release of neuropeptide Y (NPY) from nerve fibers in the myocardium reduces blood flow to the vascular tissue in the infarct area [7]. Evidence suggests that substance P (SP) has a vasodilatory effect on cardiomyocytes and a cardioprotective effect during ischemic injury [8–11]. SP reduces the likelihood of MI-induced arrhythmias, because it activates the PI3K/AKT signaling pathway and phosphorylates GSK-3, thus enhancing the expression of anti-apoptosis-related proteins and inhibiting the expression of proapoptosis proteins, thereby reducing inflammatory responses, thus protecting the heart [12]. PI3K/AKT signaling is a key regulatory pathway in the development of ischemic arrhythmias. Inhibition of this pathway causes mitochondrial damage leading to apoptosis in cardiomyocytes, and low AKT phosphorylation and high miRNA-1 levels inhibit membrane ion channel expression [12]. This changes the ion flow density, cardiac action potential duration, and cell conductivity, thereby inducing ischemic arrhythmias.

Electroacupuncture (EA) combines traditional manual acupuncture with modern electrotherapy and is now widely used to treat many conditions [13]. EA is commonly used to treat neurovascular disorders such as stroke, chronic neuropathic pain, and neurodegenerative diseases such as Alzheimer's disease [14–18]. EA exerts neuroprotective effects by enhancing anti-inflammatory response to inhibit abnormal glial cell activation and prevent neuronal loss [19]. Studies have also demonstrated that EA increases the expression of NPY in the hypothalamus and attenuates the stress response under chronic stress conditions [20, 21]. Further, EA also induces NPY expression in the paraventricular nucleus and inhibits antihypertensive and sympathetic activities [22]. EA exerts its protective effect by activating sympathetic alpha-adrenergic receptors in myocardial ischemic injury [23, 24]. EA reduces heart rate, ST segment, and infarct size, thereby alleviating myocardial injury in rats with AMI [25]. However, the mechanisms of EA in AMI treatment are largely unknown. Therefore, we speculate that EA may treat AMI by modulating neuropeptide expression.

The integration of computational techniques into traditional medicine is necessary for the integration of systems biology into traditional medicine based on a holistic approach [26–36]. In order to analyze the targets and key pathways associated with AMI treated with EA in rat models, data from the Gene Expression Omnibus (GEO) database were retrieved in this study. Moreover, neuropeptide docking with target proteins was examined. It provides new ideas for clinical treatment and drug development of AMI.

The article "Electroacupuncture Treats Myocardial Infarction by Influencing the Regulation of Substance P in the Neurovascular to Modulate PGI2/TXA2 Metabolic Homeostasis via PI3K/AKT Pathway: A Bioinformatics-Based Multiomics and Experimental Study" was retracted in 2023. Reasons: signs of a paper mill; compromised peer review; unreliable results or conclusions.

## 2. Materials and Methods

### 2.1. Patients

All patient samples were collected with informed consent in accordance with ethical standards. After blood samples were collected and centrifuged to extract serum, they were stored in ultracryogenic freezers and thawed at post-room temperatures. RNA was also extracted directly from blood cells.

### 2.2. AMI Animal Model

We purchased fifteen SPF Balb/c mice (6-week-old males) from Shanghai SLAC Laboratory Animal Co. Ltd. The mice were prebred for three days, then randomly divided into three groups; the first group was the surgical group, without ligation of the left anterior descending branch; the second group was the AMI group; and the third group was the AMI+SP group. Following shaving of the surgical scope, the surgical area was disinfected with 75% ethanol and anesthesia was administered by intraperitoneal injection with 3% sodium pentobarbital (80 mg/kg). Following anesthesia, tracheal intubation was performed to monitor the mouse's respiratory condition, and chest fluctuation was consistent with ventilator frequency (110 bpm), indicating successful intubation. With a 7-0 needle suture, mice were posed left lateral supine so their hearts were fully exposed, a little pericardium was torn, and the left anterior coronary artery descending was exposed. Afterwards, the chest was stitched layer by layer with muscles and skin. Observe the mice closely after the surgery to determine their basic health. The tracheal intubation was removed after the mice naturally awoke. Within 45 minutes after surgery, mice were injected with SP (5 nmol/kg), where the first and second groups received equal amounts of saline; about 1 week after cultivation, cardiac blood was collected, and the mice were sacrificed. Following the procedure above, mice were quickly removed, washed in ice saline to ensure no obvious blood stains, frozen at -20°C for 15 minutes, then cut into 1 mm thick slices, placed in 5 mL 1% TTC phosphate buffer (pH 7.4) and 37°C water bath for 15 minutes, and then weighed.

### 2.3. Cell Culture and RT-qPCR

DMEM high-glucose medium, supplemented with 20% FBS, 1% double antibody, and 37°C 5% CO_2_, was used to culture human cardiomyocyte (HCM) cells. Inoculation is performed at constant temperatures and humidity.

RNA extraction was performed with Trizol for cell, blood samples, and tissues, where tissue suspension was required before tissue RNA extraction, and then, Trizol was added for RNA extraction. Extracted RNA was immediately reverse transcribed into cDNA (Takara Reverse Transcription Kit) and stored at-20°C for further detection. They were thawed at room temperature, and cDNA was performed according to the RT-PCR kit of cell organisms. Among them, 2^-*ΔΔ*Ct^ calculations were performed, with GAPDH as an internal reference.

The article "Electroacupuncture Treats Myocardial Infarction by Influencing the Regulation of Substance P in the Neurovascular to Modulate PGI2/TXA2 Metabolic Homeostasis via PI3K/AKT Pathway: A Bioinformatics-Based Multiomics and Experimental Study" was retracted in 2023. Reasons: signs of a paper mill; compromised peer review; unreliable results or conclusions.

### 2.4. ELISA

NPY and SP-1 concentrations were determined using the Invitrogen ELISA kit, and human serum was diluted 100-fold. Invitrogen ELISA kit was used to determine plasma levels after centrifuging rat blood to obtain 1000-fold diluted plasma.

### 2.5. Tissue and Cellular Protein Extraction

Infarct myocardial tissue was extracted using RIPA (blue); supplemented with protease inhibitors and phosphatase inhibitors by a homogenizer (Tanon), for 30 minutes on ice; and centrifuged at 4°C 12,000 rpm for 5 min; absorbed supernatants were incubated at 100°C for 10 min, and protein denaturation was performed in a refrigerator at -20°C. Proteins were denatured at 100°C for 10 minutes and stored at -20°C after being treated with SP1 (1 mol/L and 5 mol/L) for 24 h in RIPA supplemented with protease inhibitors and phosphatase inhibitors.

### 2.6. Western Blot

Proteins were treated at different concentrations of SDS-PAGE (Yarase) and then gel electrophoresis at 10% gel at 120 V constant pressure for 100 to 120 min and 300 mA for 90 minutes; PVDF membranes were closed with 5% BSA for 1 h, blocked overnight with TBST, and the following day were incubated with the secondary antibodies for 2 h.

### 2.7. Disease-Associated Genes

We downloaded two datasets (GSE54132, GSE61840) relevant to EA treatment of MI from the NCBI GEO database (https://www.ncbi.nlm.nih.gov/geo/), and the platform annotation files were Illumina HiSeq 2000 Rat Gene expression arrays (GPL14844). Two MI rats, three EA-treated MI rats, and three normal rats are included in GSE54132; two MI rats, two EA-treated MI rats, and two normal rats are included in GSE61840.

### 2.8. DEGs Associated with EA+MI

Combining the GSE54132 and GSE61840 datasets and preprocessing (background correction, normalisation, and log2 transformation) were done with R 4.0.2 (https://www.R-project.org). Multiple probes corresponding to a common gene were averaged to determine its expression level. To eliminate batch effects between the two datasets, the “sva” package was used. DEGs with *P* < 0.05 were screened with the “limma” package, using ∣log2 fold change (FC) | ≥1.00 as the cut-off point for selecting DEGs. R software was used to plot heat maps and volcano maps related to EA+MI.

The article "Electroacupuncture Treats Myocardial Infarction by Influencing the Regulation of Substance P in the Neurovascular to Modulate PGI2/TXA2 Metabolic Homeostasis via PI3K/AKT Pathway: A Bioinformatics-Based Multiomics and Experimental Study" was retracted in 2023. Reasons: signs of a paper mill; compromised peer review; unreliable results or conclusions.

### 2.9. GO and KEGG Pathway Enrichment Analysis of DEGs

DAVID online tool was used to annotate DEGs based on GO terms. There were three categories of biological processes (BP), cellular components (CC), and molecular functions (MF) included in the GO analysis. The Kyoto Encyclopedia of Genes and Genomes (KEGG) analysis was also completed. In order to understand the specific mechanisms of EA treatment of MI, we used the pathview-Bioconductor software (version 3.15) package to map signaling pathways.

### 2.10. Protein and Neuropeptide Docking

Peptide-core protein docking was performed between SP and the receptor protein to investigate their interaction. By homology modeling and exporting the 3D structure to PDB, we constructed SP's sdf structure from the PubChem database. We first downloaded the PDB format of the receptor core protein from the PDB website (http://www.rcsb.org/), dehydrated and dephosphorylated the protein using PyMOL software, and converted the SP and core protein structural domains to the PDBqt format using AutoDockTools 1.5.6 software. In order to calculate the molecular binding energy and show the results of molecular docking, the Vina script was run. The binding energy of a ligand and receptor can be less than zero, and spontaneous binding can take place. Vina binding energies ranging from -5.0 kcal/mol are used to evaluate the accuracy of bioinformatics predictions for ligand-receptor complexes.

### 2.11. Statistical Method

All experiments were performed three times. The data are presented as mean ± SD (standard deviation). Chi-square tests were used to analyze frequency differences between two groups, and *t*-tests were used to analyze differences between independent samples. *P* < 0.05 was considered statistically significant.

## 3. Results

### 3.1. SP Expression Was Increased in AMI Patients

Neuropeptides play roles in numerous diseases. Therefore, to investigate the role of SP in AMI, we collected blood from patients with AMI, and the expression of the neuropeptides was measured using RT-qPCR. Compared to the normal population, an increase in expression of SP, angiotensin II (Ang II), and NPY was observed in the serum of AMI patients. Among these, there was a significant increase in SP levels in AMI patients (Figure 1(a)). ELISA results revealed that as compared to the normal population, no significant difference (*P* > 0.001) in NPY levels was observed in the serum of AMI patients (Figure 1(b)). AMI patients' serum SP levels were significantly higher than those in the normal population, as shown in Figure 1(c) (*P* < 0.001). The results of this study indicate a significant increase in SP levels in AMI patients; however, its role in the disease is unclear.

The article "Electroacupuncture Treats Myocardial Infarction by Influencing the Regulation of Substance P in the Neurovascular to Modulate PGI2/TXA2 Metabolic Homeostasis via PI3K/AKT Pathway: A Bioinformatics-Based Multiomics and Experimental Study" was retracted in 2023. Reasons: signs of a paper mill; compromised peer review; unreliable results or conclusions.

### 3.2. Mice with AMI Can Benefit from SP

To investigate the effect of SP on acute MI, we established a mouse model of acute MI by ligation of the left anterior coronary artery descending and observed the effect of SP on AMI (Figure 2(a)). We used myocardial infarcted mice as control groups, and the SP-acting mice had both decreased infarct area weight and infarct tissue proportion (infarcted myocardial weight/total heart weight), indicating that SP was protective against AMI (Figures 2(b) and 2(c)).

### 3.3. SP Influences PGI2/TXA2 Axis Balance by Altering the PI3K/AKT Pathway

Our results show a protective effect of SP on AMI; however, SP's mechanism of action on AMI is unclear. In addition to the rupture of coronary artery plaque to form a clot that blocks the lumen of the artery, an increase in oxygen consumption by the myocardium and coronary artery spasm can also induce AMI [1, 2]. Coronary spasms are caused by various factors, like prostacyclin (PGI2) and thromboxane A2 (TXA2) [3, 4]. Therefore, ELISA was used to check the protein levels of PGI2 and TXA2 in the sera of the mice. As shown in Figures 3(a) and 3(b), as compared to normal mice, the levels of PGI2 and TXA2 were elevated in acute MI mice. Further, compared to the control group, the levels of PGI2 were higher in SP-treated MI mouse models. However, compared to the control group, a decrease in the levels of TXA2 was observed in SP-treated MI mouse models. Therefore, we hypothesized that SP affected MI by altering PGI2/TXA2 balance.

In the SP group, *Pik3ca*, *Akt*, and *Mtor* gene expression was increased, as shown in Figure 3(c). Therefore, we hypothesized that the PI3K/AKT pathway was involved in the mechanism of action of SP in AMI. We used western blotting to determine the expression of AKT, p-AKT, and mTOR proteins. The results reveal an increase in AKT, p-AKT, and mTOR expression in AMI mice treated with SP compared to the control (Figure 3(d)).

To further analyze the mechanism of action of SP on cardiomyocytes, the human cardiomyocyte cell line HCM was treated with SP. RT-qPCR results revealed an increase in the expression of PI3K pathway-related genes (*Pik3ca*, *Pik3cb*, *Akt*, and *Mtor*) in HCM cells treated with SP (Figure 3(e)) compared to untreated HCM cells. The protein expression of these genes, as confirmed by western blotting, was consistent with RT-PCR results. Therefore, it is tempting to conclude that SP promotes AKT, p-AKT, and mTOR expression in cardiomyocytes (Figure 3(f)). Taken together, we show that SP influences the PGI2/TXA2 hemostasis by the PI3K/AKT pathway, thereby alleviating the symptoms of AMI.

### 3.4. Gene Expression Analysis of MI-Related Genes Treated with EA

GSE54132 and GSE61840 datasets were retrieved from the GEO database. The datasets used the same platform (GPL14844, Illumina HiSeq 2000 array) for the high-throughput mRNA sequencing of the EA-treated MI rat model. The gene expression was normalized after preprocessing and background correction. Differentially expressed genes (DEG) were screened using linear models for microarray data (limma) package. There were 551 DEGs between the MI rat model and control rats, of which 346 were expressed upregulated while 205 were expressed downregulated. However, in EA-treated MI rats, a total of 541 DEGs were observed, of which 197 were upregulated, and 344 were downregulated. The top 100 genes with the highest expression in MI-CTR (control) and EA-treated MI rats were screened for hierarchical cluster analysis, and the cluster heat map (Figures 4(a) and 4(c)) and volcano map (Figures 4(b) and 4(d)) were constructed. Differential expression of *Myd88*, *Mtor*, *Akt1*, *Sp*, and *Irak1* was observed between MI-CTR and EA-treated MI rats, consistent with the experimental results. There was no significant difference in the expression profile of other genes.

The article "Electroacupuncture Treats Myocardial Infarction by Influencing the Regulation of Substance P in the Neurovascular to Modulate PGI2/TXA2 Metabolic Homeostasis via PI3K/AKT Pathway: A Bioinformatics-Based Multiomics and Experimental Study" was retracted in 2023. Reasons: signs of a paper mill; compromised peer review; unreliable results or conclusions.

### 3.5. DEG Related to EA-Treated MI

The VennDiagram R package was used to reduplicate the intersection of DEG in MI-CTR and EA-treated MI [37]. The results reveal 135 DEGs, of which 119 were upregulated and 16 were downregulated in MI. In the EA-treated MI model, 16 genes were upregulated, and 119 were downregulated. There was an inverse correlation between DEG on the MI-CTR and EA-treated MI group. This indicates that EA treatment significantly reversed the expression of DEG in MI compared to the control group. Therefore, all 135 DEGs could be used as a potential target for EA treatment of MI (Figure 5).  Table 1 shows the expression of the specific gene targets validated in the previous experiments in the MI-CTR and EA-treated MI groups.

### 3.6. GO and KEGG Pathway Enrichment Analysis of DEGs

The Database for Annotation, Visualization and Integrated Discovery (DAVID) was used for data processing and analysis, and *P* < 0.05 was used as a criterion selection of genes for enrichment analysis. Gene Ontology (GO) analysis revealed 135 DEGs and the biological processes, including positive regulation of tumor necrosis factor production, tumor necrosis factor superfamily cytokine production, cellular responses to oxidized low-density lipoprotein (LDL) particle stimulation, carboxylic acid transaminase, stimulation of LDL particles, carboxylic acid transmembrane transport, and organic acid transmembrane transport. Molecular functions include neutral amino acid transmembrane transporter activity, amino acid transmembrane transporter activity, alanine, carboxylic acid, and organic acid transmembrane transporter activity. The cellular components enriched were late endosomal membranes, lysosomal membranes, lysosomal vacuolar membranes, proton-transporting V-type ATPase complex AB, and the transcriptional regulator complex (Figures 6(a) and 6(b)). Pathway enrichment analysis was performed using the Kyoto Encyclopedia of Genes and Genomes (KEGG) database (Figure 6(c)). KEGG pathway analysis of 135 DEGs mainly enriched the NF-*κ*B signaling pathway, collecting ductal acid secretion, steroid hormone biosynthesis, rheumatoid arthritis, PI3K/AKT signaling pathway, etc. The pathview-Bioconductor software (version 3.15) was used to show the potential signaling pathways associated with EA treatment of MI (Figure 6(d)).

The article "Electroacupuncture Treats Myocardial Infarction by Influencing the Regulation of Substance P in the Neurovascular to Modulate PGI2/TXA2 Metabolic Homeostasis via PI3K/AKT Pathway: A Bioinformatics-Based Multiomics and Experimental Study" was retracted in 2023. Reasons: signs of a paper mill; compromised peer review; unreliable results or conclusions.

### 3.7. SP-Core Protein Docking

Linear structure modeling was performed on the neuropeptide amino acid sequence and exported in PDB format. Three dimensional (3D) structures of the core proteins MYD88, IRAK1, NFKB1, PIK3CA, AKT1, and MTOR were downloaded from the PDB database and exported in PDB format, and SP as the core structural domain was converted using AutoDockTools 1.5.6 software. The results reveal that the binding energies of the core proteins PIK3CA, AKT1, and mTOR to SP were below -5.0 kcal/mol, and the Root Mean Square Deviation (RMSD) was <5.00 (Table 2). Combining the RMSD, chemical energy and docking model, the core protein AKT1 formed the most stable docking bond with SP. Finally, the results were exported using Vina and PyMOL, and the 3D molecular docking with protein ligands was demonstrated using Discovery Studio 2019 software (Figure 7) (Table 2).

## 4. Discussion

Substance P (SP) is a tachykinin located mainly in the sensory nerves and abundantly found in the cerebrum and intestinal region. It is widely distributed in the central nervous system and gastrointestinal system. It has nociceptive transmission, participates in the inflammatory response and immune regulation, and affects reproductive endocrine functions. In the heart, SP is usually located in the coronary artery [38–40]. To a lesser extent, the peripheral sensory nerves are located in coronary endothelial cells [41]. Thus, SP is a modulator of perception and released in response to changes in coronary blood flow or pressure, such as during myocardial ischemia [42]. SP is released within a minute of ischemic injury [41], and SP level remains elevated even during the reperfusion phase [10]. There is substantial evidence that SP has a cardioprotective effect in ischemic injury by mediating potent coronary dilatory effect on cardiomyocytes [8–11]. SP acts as an immunomodulator by binding to the neurokinin-1 receptor (NK-1R). NK-1R antagonism inhibits the beneficial effects of SP in restoring contractile function and coronary blood flow. In mouse isolated perfusion heart model, NK-1R blocking resulted in increased left ventricle (LV) diastolic blood pressure (DBP) and decreased systolic function. In contrast, adding exogenous SP decreased LV DBP and improved systolic function, suggesting that exogenous SP could also provide additional protective effects over endogenous SP [8, 10].

The article "Electroacupuncture Treats Myocardial Infarction by Influencing the Regulation of Substance P in the Neurovascular to Modulate PGI2/TXA2 Metabolic Homeostasis via PI3K/AKT Pathway: A Bioinformatics-Based Multiomics and Experimental Study" was retracted in 2023. Reasons: signs of a paper mill; compromised peer review; unreliable results or conclusions.

EA has a protective role in myocardial ischemic injury [23, 24]. EA reduces heart rate, ST segment, and MI area and alleviates myocardial injury in rats with AMI [25]. EA may also have a beneficial effect on ischemic heart disease such as MI by reducing lipid peroxidation; promoting energy metabolism, myocardial oxygen demand, and myocardial enzyme activity; and altering cellular ultrastructure. However, its mechanism of action is not yet clear [43–45].

Various studies have shown that the mechanism of EA treatment is closely related to SP. The SP-mediated pathway may be involved in the analgesic effect of EA in rats. Studies have shown that inhibiting the SP signaling can significantly enhance the analgesic effect of EA [46, 47]. EA may also improve gastrointestinal symptoms by reducing the SP expression in the colonic mucosa of patients with irritable bowel syndrome [48]. Additionally, in hypertension or colitis rat models, increased SP expression at acupoints leads to neurogenic inflammation, extravasation of plasma, and accumulation of subcutaneous water content. This results in high conductance and low impedance, triggering acupuncture signaling [49, 50]. Elevated SP levels also increase the therapeutic effect of EA [51, 52]. Consistent with previous studies, our results reveal that SP was differentially expressed in MI-CTR and EA-treated MI rat models, suggesting that SP may be involved in the effect of EA treatment on AMI.

Several studies have shown that EA mediates its effect via the PI3K/AKT pathway. EA significantly activates the PI3K/AKT signaling pathway in ischemic brain tissue, thereby exerting a neuroprotective effect in ischemic stroke, thus improving learning and memory function in a cerebral ischemia/reperfusion injury animal model [53, 54]. EA ameliorates denervation-induced skeletal muscle atrophy in rats via the PI3K/AKT signaling pathway [55]. In addition, EA reduces pulmonary vascular remodeling in the COPD model via the PI3K/AKT signaling pathway. In spontaneously hypertensive rats, EA reduces phenotypic transformation of vascular smooth muscle cells via the PI3K/AKT signaling pathway [56, 57]. Our results reveal that AKT and PIK3CA expression was upregulated in AMI myocardial tissues and that AKT1 was differentially expressed in MI-CTR and EA-treated MI rats. Therefore, EA may play a therapeutic role in AMI via the PI3K/AKT pathway.

The article "Electroacupuncture Treats Myocardial Infarction by Influencing the Regulation of Substance P in the Neurovascular to Modulate PGI2/TXA2 Metabolic Homeostasis via PI3K/AKT Pathway: A Bioinformatics-Based Multiomics and Experimental Study" was retracted in 2023. Reasons: signs of a paper mill; compromised peer review; unreliable results or conclusions.

PGI2/TXA2, a vasomodulator, was also involved in the EA's mechanism of action. Acute alcoholic liver injury animals showed higher levels of the vasoconstrictor TXA2 and decreased levels of the vasodilator PGI2; EA stimulation partially restored levels of PGI2/TXA2 in liver tissue [58]. EA also affects vascular function in various diseases, including vascular dementia, by reducing vascular hyporesponsiveness in a portal hypertension rat model [25, 59]. The dynamic homeostasis of PGI2/TXA2 is essential in maintaining normal vascular tone and patency, and an elevated ratio is associated with atherosclerosis [60]. Consistent with the previous studies, we report that both PGI2 and TXA2 levels were elevated in the AMI mouse model and the involvement of PGI2/TXA2 in the effect of EA treatment on AMI.

Atherogenesis is caused by a buildup of PGI2 in the body, which inhibits TXA2, an arachidonic acid metabolite implicated in platelet aggregation [61]. TXA2 is released by cardiac muscle under hypoxia and early reoxygenation conditions [62, 63], and cardiac-derived TXA2 could be responsible for initiating the reperfusion injury in the heart [64]. Prostacyclin (PGI2) is an endogenous prostaglandin formed and released by endothelial cells with antiplatelet, vasodilatory, and cytoprotective properties [65]. PGI2 can also inhibit endothelial cell apoptosis and decomposition, which protects vascular integrity [66]. Due to vasodilatory properties, PGI2 is currently used in treating pulmonary hypertension and critical limb ischemia [67, 68]. It has been shown that patients after coronary stenting treated with low-dose prostacyclin have improved endothelial function due to reduced levels of the soluble endothelial biomarker, sE-selectin. In this study, PGI2 and TXA2 were elevated in mice with AMI compared with normal mice. Further, in the SP-treated AMI mouse model, the levels of PGI2 were higher than in the control mice. Compared to the control group, a decrease in TXA2 levels was observed in the SP-treated AMI mouse model. Therefore, it is likely that SP may have a protective effect on AMI by altering the balance of PGI2/TXA2.

In this study, upregulation in the expression of PI3K pathway-related genes, including *Pik3ca*, *Akt*, and *Mtor*, was observed in infarcted myocardial tissue of mice by RT-PCR. Western blotting results reveal an increase in expression of AKT, p-AKT, and MTOR in AMI treated with SP. Further, human cardiomyocyte cells (HCM) treated with SP increased mRNA and protein expression of PI3K/AKT pathway-related genes (PIK3CA, PIK3CB, AKT, and MTOR). In addition, analysis of high-throughput sequencing data retrieved from the GEO database showed a differential expression of *Myd88*, *Mtor*, *Akt1*, *Sp*, and *Irak1* in MI-CTR and EA-treated MI rat models. These results were consistent with the in vivo and in vitro studies, while the remaining genes showed no significant differences. KEGG analysis of DEG in EA-treated MI tissues showed significant enrichment of the PI3K/AKT signaling pathway. Molecular docking analysis also confirmed that core proteins PIK3CA, AKT1, and MTOR formed stable docking bonds with SP with binding energies below -5.0 kcal/mol. The core protein AKT1 formed the most stable docking model with SP. Therefore, we postulate that SP promotes the expression of AKT, p-AKT, and MTOR in cardiomyocytes, thereby improving cardiomyocyte survival via NK-1R activation. Our study is based on previous reports and clinical data, validated by in vivo and in vitro studies. However, the number of clinical samples was limited and requires further in vivo validations.

The article "Electroacupuncture Treats Myocardial Infarction by Influencing the Regulation of Substance P in the Neurovascular to Modulate PGI2/TXA2 Metabolic Homeostasis via PI3K/AKT Pathway: A Bioinformatics-Based Multiomics and Experimental Study" was retracted in 2023. Reasons: signs of a paper mill; compromised peer review; unreliable results or conclusions.

## 5. Conclusion

EA regulates PGI2/TXA2 metabolism directly or indirectly through SP to reduce myocardial cell injury and alleviate the symptoms of AMI by affecting PI3K/AKT pathway activity. It provides an idea for clinical drug research and development.

## Figures and Tables

**Figure 1:** SP expression is increased in AMI patients. (a) RT-PCR showed that SP, Ang II, and NPY were increased in AMI patients. (b) ELISA results show NPY levels in the serum of AMI patients. (c) ELISA results reveal higher levels of SP in the serum of AMI patients. ^∗^*P* < 0.05, ^∗∗^*P* < 0.01, and ^∗∗∗^*P* < 0.001.

**Figure 2:** SP can improve the symptoms in the AMI mouse model: (a) schematic representation of the AMI mouse model; (b) the weight of infarcted myocardium (45 min); (c) the weight of infarcted myocardium (7 d); ^∗^*P* < 0.05.

**Figure 3:** SP affects the PGI2/TXA2 balance by influencing the PI3K/AKT pathway. (a) Determination of PGI2 concentrations in mouse serum by ELISA; (b) determination of TXA2 concentrations in mouse serum by ELISA; (c) RT-PCR of *Myd88*, *Irak1*, *Tab1*, *Nf-κb1*, *Pik3c1*, *Akt*, and *Mtor* gene expression in infarcted myocardial tissues of mice; (d) expression of MTOR, p-AKT, AKT, and GAPDH genes in infarcted myocardial tissues of mice by western blot; (e) expression of *Myd88*, *Irak1*, *Tab1*, *Nf-κb1*, *Pik3c1*, *Akt*, and *Mtor* genes after SP treatment; (f) expression of MTOR, p-AKT, AKT, and MTOR after SP treatment by western blot.

The article "Electroacupuncture Treats Myocardial Infarction by Influencing the Regulation of Substance P in the Neurovascular to Modulate PGI2/TXA2 Metabolic Homeostasis via PI3K/AKT Pathway: A Bioinformatics-Based Multiomics and Experimental Study" was retracted in 2023. Reasons: signs of a paper mill; compromised peer review; unreliable results or conclusions.

**Figure 4:** DEGs associated with EA+MI based on microarray data. (a) Heat map of MI-CTR differentially expressed genes; (b) heat map of MI-CTR differentially expressed volcanoes; (c) heat map of EA+MI differentially expressed genes; (d) heat map of EA+MI differentially expressed volcanoes. Blue represents ascending genes; red represents descending genes. Genes marked with an asterisk have been validated in the current experiment.

**Figure 5:** Venn diagram showing EA treatment targets for MI.

**Figure 6:** DEG enrichment analysis using GO and KEGG. (a) GO functional analysis bubble diagram; (b) GO functional analysis histogram; (c) KEGG functional analysis bubble diagram; (d) PI3K/AKT signaling pathway.

**Figure 7:** Molecular docking model of neuropeptide SP-core protein, Myd88-substance P-3D (a), Irak1-substance P (b), Nfkb1-substance P (c), Pik3ca-substance P-3D (d), AKT1-substance P (e), and MTOR-substance P (f).

**Table 1:** Target expression in MI-CTR and EA+MI.

Gene symbol (Rattus norvegicus)	MI-CTR		EA+MI	
	log_2_FC	*P* value	log_2_FC	*P* value
Myd88	3.54	*P* < 0.001	-2.85	0.003
MTOR	6.26	*P* < 0.001	-6.68	*P* < 0.001
AKT1	6.06	0.003	-5.80	0.003
SP	1.79	0.016	-2.74	0.003
Irak1	1.69	0.025	-2.18	0.042

**Table 2:** Docking results for neuropeptide SP with core proteins using AutoDock Vina.

Protein	Compound	Structure	Vina (kcal·mol^−1^)	RMSD
Myd88 (5AIU)	Substance P		-1.5	0
Irak1 (6BFN)	Substance P		-4.4	2.372
Nfkb1 (5LW1)	Substance P		-4.5	0
Pik3ca (5SX8)	Substance P		-8.4	2.029
AKT1 (4EJN)	Substance P		-8.5	1.315
Mtor (2L0X)	Substance P		-5.4	3.0

## Data Availability

This study's raw data can be downloaded from the database, and the experimental data can be obtained from the corresponding authors.
